# Properly Folded Bacterially Expressed H1N1 Hemagglutinin Globular Head and Ectodomain Vaccines Protect Ferrets against H1N1 Pandemic Influenza Virus

This article has been retracted.

**DOI:** 10.1371/journal.pone.0011548

**Published:** 2010-07-12

**Authors:** Surender Khurana, Swati Verma, Nitin Verma, Corey J. Crevar, Donald M. Carter, Jody Manischewitz, Lisa R. King, Ted M. Ross, Hana Golding

**Affiliations:** 1 Division of Viral Products, Center for Biologics Evaluation and Research (CBER), Food and Drug Administration (FDA), Bethesda, Maryland, United States of America; 2 Center for Vaccine Research, University of Pittsburgh, Pittsburgh, Pennsylvania, United States of America; Institute of Molecular and Cell Biology, Singapore

## Abstract

**Background:**

In the face of impending influenza pandemic, a rapid vaccine production and mass vaccination is the most effective approach to prevent the large scale mortality and morbidity that was associated with the 1918 “Spanish Flu”. The traditional process of influenza vaccine production in eggs is time consuming and may not meet the demands of rapid global vaccination required to curtail influenza pandemic.

**Methodology/Principal Findings:**

Recombinant technology can be used to express the hemagglutinin (HA) of the emerging new influenza strain in a variety of systems including mammalian, insect, and bacterial cells. In this study, two forms of HA proteins derived from the currently circulating novel H1N1 A/California/07/2009 virus, HA1 (1–330) and HA (1–480), were expressed and purified from *E. coli* under controlled redox refolding conditions that favoured proper protein folding. However, only the recombinant HA1 (1–330) protein formed oligomers, including functional trimers that bound receptor and caused agglutination of human red blood cells. These proteins were used to vaccinate ferrets prior to challenge with the A/California/07/2009 virus. Both proteins induced neutralizing antibodies, and reduced viral loads in nasal washes. However, the HA1 (1–330) protein that had higher content of multimeric forms provided better protection from fever and weight loss at a lower vaccine dose compared with HA (1–480). Protein yield for the HA1 (1–330) ranged around 40 mg/Liter, while the HA (1–480) yield was 0.4–0.8 mg/Liter.

**Conclusions/Significance:**

This is the first study that describes production in bacterial system of properly folded functional globular HA1 domain trimers, lacking the HA2 transmembrane protein, that elicit potent neutralizing antibody responses following vaccination and protect ferrets from *in vivo* challenge. The combination of bacterial expression system with established quality control methods could provide a mechanism for rapid large scale production of influenza vaccines in the face of influenza pandemic threat.

## Introduction

In April 2009, the Centers for Disease Control and Prevention (CDC) announced the detection of a novel strain of influenza virus in humans. The novel virus derived its genes from viruses circulating in the pig population [1], [2], [3]. Due to sustained human-to-human transmission of this novel virus throughout the world, on June 11^th^ the World Health Organization (WHO) raised the worldwide pandemic alert level to Phase 6.

The most effective way to curtail pandemics is by mass vaccination [4], [5]. At the moment there are two types of licensed vaccines against seasonal influenza in the US: subunit (split) inactivated vaccines (IV) and live cold adapted attenuated influenza vaccine (LAIV) [6] [7], [8]. Both vaccines are grown in chicken eggs. The process of constructing a new vaccine strain based on newly circulating viruses is quite lengthy. It involves in vivo (in chicken eggs) or *in vitro* (in cell culture using reverse genetics techniques) reassortment between the internal genes of a donor virus such as A/PR/8/34 with the hemagglutinin (HA) and neuraminidase (NA) of the new influenza strain. The candidate vaccine strains must be further selected based on their high growth capability in eggs before they can be used for production of vaccines. Moreover, the manufacturing process is limited in scalability by the use of eggs and the amount of purified virus that can be produced. This process is used for the production of seasonal influenza vaccines every year, but it may pose a clear impediment to initiation of rapid mass vaccination against spreading pandemic influenza, as was evident for the 2009 H1N1 virus.

Recombinant HA based vaccines provide an alternative that could save several months of manufacturing time, since the HA gene of the newly circulating strain is available shortly after virus isolation. Expression of HA in insect cells and mammalian cells are under development and/or clinical trials [9], [10], [11]. The main challenge to the recombinant technology is to ensure that the HA products resemble the native virion-associated trimeric spike proteins and can elicit robust immune responses targeting protective conformational epitopes in the globular domain of HA.

In previous studies, we constructed H5N1 whole-genome-phage-display libraries (GFPDL) and used them to map the antibody responses following human infection with highly pathogenic H5N1 (A/Vietnam/1203/2004), as well as post-H5N1 vaccination sera. We identified large HA1 fragments, encompassing the receptor binding domain (RBD), that were bound by broadly neutralizing human monoclonal antibodies from H5N1 recovered individuals and by polyclonal convalescent sera. Several HA1 fragments were expressed and purified from *E. coli* inclusion bodies, and were shown to be properly folded and presented conformational epitopes [12]. The bacterially expressed HA1 proteins were also shown to absorb most of the neutralizing activity in post-H5N1 infection and post-H5N1 vaccination sera [12], [13]. Based on these studies, it was predicted that HA1 fragments that contain most of the neutralizing antibody targets may generate protective immunity against emerging influenza strains.

Compared with insect or mammalian cells, expression of recombinant proteins in bacteria could present a viable alternative in terms of large scale vaccine production and a short time line suitable for rapid response in influenza pandemic. Several studies with bacterially expressed HA proteins based on the H5N1 avian influenza virus (AIV) were reported [14], [15], [16], and one clinical trial with a bacterially expressed fusion protein between the HA fragment and flagellin from *Salmonella typhimurium* type 2 (STF2), a TLR5 agonist is underway [17]. However, bacterially expressed HA proteins are not subjected to the post-translational modifications that takes place in eukaryotic cells, including step-wise glycosylation process important for proper folding of the HA protein, as well as trimerization and transport to the cell membrane [18], [19], [20]. Indeed it was argued that in the absence of glycosylation, the newly synthesized HA proteins are not likely to fold properly or trimerize like native HA molecules, and may not present native conformational epitopes, which are important for generation of an effective protective immune response. Indeed the majority of the previous studies did not demonstrate proper folding and/or oligomerization of the HA proteins produced in prokaryotic systems [14], [15], [16], [21], [22]. To address this concern, we established multiple assays to monitor the integrity of bacterially expressed HA proteins for proper folding, formation of trimers and oligomers, receptor binding, and agglutination of red blood cells (RBC). Here, we describe the properties of two novel H1N1 swine-like HA proteins, HA1 (1–330) and HA (1–480), expressed in *E. coli.* Both proteins were properly folded as determined by CD spectra, binding to post-infection and post-vaccination sera, and could adsorbed neutralizing activity from H1N1 immune sera. However, only the bacterially expressed HA1 globular domain (1–330) contained functional trimers and oligomers capable of receptor binding and RBC agglutination. Importantly, vaccination of ferrets with both proteins resulted in reduced viral loads in nasal washes following challenge with novel H1N1 A/California/07/2009. However, after low dose vaccination (important for dose-sparing in pandemic scenario), HA1 (1–330) provided better reduction of morbidity (body temperature elevation and weight loss) compared with HA (1–480) *in vivo.*

## Results

### Properties of bacterially expressed H1N1 HA1 (1–330) and HA (1–480)

DNA fragments encoding amino acid sequence 1–330 and 1–480 of HA from A/California/07/2009 were cloned as *NotI-PacI* inserts in the T7 promoter based expression vector with His_6_ tag at the C-terminus [13]. Both fragments of H1N1 HA expressed in *E. coli* Rosetta Gami cells (Novagen) localized to insoluble fraction (inclusion bodies). IBs were refolded *in vitro* under controlled redox conditions and purified by HisTrap Fast flow chromatography. This process was previously shown to generate highly purified properly folded HA1 fragments from H5N1 [13]. The purified HA1 (1–330) and HA (1–480) proteins ran as a single band on SDS-PAGE with the anticipated MW of approximately 30 and 50 kDa, respectively (Fig. 1A).

**Figure 1:** Biochemical and functional characterization of bacterially expressed and purified H1N1 HA proteins. (A) Purified *E. coli* derived HA proteins were analyzed by SDS-PAGE. DNA encoding HA1 (1–330) and HA (1–480) from HA gene segment of A/California/07/2009 (H1N1) generated from egg-grown virus were used for cloning in a T7 promoter based expression vector (pSK) where the desired polypeptide can be expressed as fusion protein with His_6_ tag at the C-terminus. The proteins were expressed, denatured and refolded under controlled redox conditions and purified using His-Trap fast flow chromatography to >90% purity (see Materials and Methods). The purified proteins run at their corresponding molecular weight in reducing SDS-PAGE. (B-C) CD melt spectroscopy shows that both H1N1 HA1 (1–330) (B) and H1N1 HA (1–480) (C) are properly folded. Both H1N1 HA proteins, at a concentration of 0.5 mg/ml in 20 mM PBS, pH 7.2, were subjected to heating at 0.5°C/min increments. The protein unfolding kinetics was measured at 222 nm using a J-715 Circular Dichroism system (JASCO corp., Easton, MD). (D-E) Superdex S-200 gel filtration chromatography of purified H1N1 HA proteins from *E.coli*. The panels present superimposed elution profiles of purified HA proteins (red line) overlaid with calibration standards (grey line). (D) The H1N1 HA (1–330) protein purified from bacterial cells existed as approximately 20% high-molecular-mass oligomer (>600 kDa), 45% trimer (∼110 kDa) and 35% monomer (34kDa) (red line). (E) H1N1 HA (1–480) is present only as a monomer (50kDa). (**F-G**) **Binding kinetics of purified H1N1 HA proteins in a SPR based receptor binding assay.** Steady-state equilibrium analysis of different H1N1-HA proteins to fetuin and its asialylated counterpart (Asialo-fetuin) was analyzed at 25°C using a ProteOn surface plasmon resonance biosensor (BioRad Labs). Samples of purified H1N1-HA proteins (10 µg/ml) were injected simultaneously over a mock surface to which no protein was bound, followed by the Asialofetuin in (F) or Fetuin in (G) immobilized on a sensor chip through the free amine group, and onto a blank flow cell, free of protein. Binding kinetics and data analysis were performed using ProteOn system surface plasmon resonance biosensor instrument (BioRad Labs, Hercules, CA). (H) Agglutination of human RBCs by properly folded bacterial H1N1 HA (1–330) protein. Serial dilutions of purified HA proteins or virus were mixed with washed RBC and incubated to analyze the receptor binding and cross-linking of human RBC. Virus H1N1xPR8 A/California/07/2009 (X-179A) was used as a control. Strong hemagglutination was observed for bacterial H1N1 HA (1–330) but not with either bacterial H1N1 HA (1–480) or mammalian H1N1 HA0.

To determine if the bacterially expressed (unglycosylated) HA1 (1–330) and HA (1–480) proteins are properly folded they were analyzed by CD spectroscopy. The change in elipticity at 222 nm, which monitors unfolding of α-helix structures over a range of temperatures (CD melt), confirmed that both HA1 (1–330) and HA (1–480) behaved as properly folded proteins with a melting temperature around 52°C (Fig. 1 B-C).

We next determined if the bacterially expressed proteins oligomerized into higher molecular forms, using gel filtration chromatography on Superdex S200 XK 16/60 column (GE-Healthcare). Surprisingly, the HA1 (1–330) protein contained at least 50% of trimers and oligomers (Fig. 1D), while the larger HA (1–480) contained only monomers (Fig. 1E). To further investigate which HA forms are required for receptor binding we established a fetuin based SPR assay that mimics the simultaneous interactions between the virion spikes and multiple sialic acid moieties[23]. The bacterially expressed HA1 (1–330), HA (1–480), and a mammalian cell derived recombinant full length HA (HA0) (from Immune Technology Corp, NY) were tested for binding to fetuin coated on biosensor chips. As shown in Fig. 1G, only HA1 (1–330) bound efficiently to fetuin (but not to asialo-fetuin; Fig. 1F). In contrast, neither the mammalian cell derived HA0, nor the bacterially expressed HA (1–480) proteins bound to the fetuin in SPR (Fig. 1G).

In addition to receptor binding, hemagglutination of red blood cells (RBC) is a surrogate assay to measure the functionality of the influenza hemagglutinin. The presence of trimers and oligomers (mimicking the virion spikes) is required for the formation of RBC lattice [24]. As seen in Fig. 1H, H1N1 virions (positive control) agglutinated RBC very well at all the dilutions used. Bacterially expressed H1N1 HA1 (1–330) protein (containing trimers and oligomers) also agglutinated human RBC very efficiently, even at the lowest concentration of 45 ng/ml. On the other hand, the bacterially expressed HA (1–480) and mammalian cell derived recombinant HA0 did not agglutinate human RBC. These differences in hemagglutination were in agreement with the results obtained in the fetuin binding SPR assay. The lack of agglutinating capacity most likely reflected the absence of stable trimers and oligomers in the HA (1–480) or the mammalian cell derived HA0 protein preparations.

### Bacterially expressed H1N1 HA (1–330) and HA (1–480) and mammalian-expressed HA0 are recognized by sera from ferrets infected with A/California/07/2009 and post vaccination human sera

The differences in the functional properties of HA1 (1–330) compared with the larger proteins containing the HA1+HA2 ectodomain needed further investigation. It was important to confirm that all three proteins expressed conformational “native” antigenic epitopes, recognized by antibodies elicited by H1N1 infection or by immunization with traditional (inactivated) vaccine. Ferrets are a good animal model for influenza virus pathogenesis. Following H1N1 infection, ferrets undergo transient loss of body weight, elevation in body temperature, and extensive viral replication in the upper and lower respiratory track on days 1–5, followed by viral clearance and recovery between Days 7–14 [25]. In the current study, consecutive post-H1N1 infection sera were evaluated for virus neutralizing antibody titers in a microneutralization assay (MN) (Fig. 2A) and for binding to recombinant H1N1 HA proteins by surface plasmon resonance (SPR), using either mammalian cell expressed HA0 or the bacterially expressed H1N1 HA1 (1–330) and HA (1–480) proteins (Fig. 2B–D). MN titers in the ferret sera were <20 during the first 5 days, followed by a rapid rise on days 7 and 14, and started to decline there after (Fig. 2A). On the other hand, using SPR, HA binding antibodies were measured as early as day 5 post infection and peaked on day 14. Importantly, binding of post-H1N1 infection ferret sera to HA0 from mammalian cells and to the bacterially expressed HA1 (1–330) and HA (1–480) proteins demonstrated similar kinetics and binding avidity profiles (Fig. 2 B-C-D), confirming that the bacterially expressed proteins were antigenically similar to the mammalian cell derived HA. The significant increase in binding to H1N1-HA proteins on days 7 and 14 correlated with the appearance of neutralizing antibodies against A/California/07/2009 (Fig. 2A). We also evaluated the binding of pre-and post-vaccination sera from two individuals that were immunized with a licensed inactivated subunit A/California/7/2009 vaccine (Fig. 2 E-F-G). Post-vaccination sera bound to mammalian-expressed HA0 (Fig. 2E) and to bacterially-expressed HA1 (1–330) (Fig. 2F) & HA (1–480) (Fig. 2G) proteins. The SPR results confirmed that all three proteins were properly folded and expressed native conformational epitopes. Interestingly, in both ferret and human studies, antibody binding to the HA1 (1–330) (containing trimers) was superior to that observed with the mammalian cell derived HA0 and the bacterially expressed HA ectodomain proteins (Fig. 2C vs. 2B and 2D, and Fig. 2F vs. 2E and 2G).

**Figure 2:** Development of neutralizing and anti-HA binding antibodies following wt H1N1 (A/California/7/2009) infection in ferrets & post-H1N1 vaccination (inactivated vaccine) in humans. (A) **Microneutralization of H1N1 A/California/2009 virus with post-H1N1-infected ferret samples.** End-point titers (mean of three replicates) using post-infection sera from multiple ferrets at each time point in a microneutralization assay performed with A/California/07/2009 (X-179A). For day 21, sera of ten animals were pooled. Each dot in other time-points represents an individual H1N1 infected ferret. (B–D) **Antibody kinetics following H1N1 challenge in ferrets.** Steady-state equilibrium analysis of post-H1N1 infected ferret sera or pre- & post-H1N1 vaccinated human sera to mammalian H1N1 HA0 (Immune Technologies, NY) and properly folded bacterially expressed H1N1 HA1 (1–330) or H1N1 HA (1–480) fragment were measured using SPR. Ten-fold diluted individual post-infection sera from each time point, were injected simultaneously onto recombinant mammalian H1N1 HA0 in (B) and properly folded bacterially expressed H1N1 HA1 (1–330) in (C) or H1N1 HA (1–480) in (D), immobilized on a sensor chip through the free amine group, and onto a blank flow cell, free of peptide. SPR binding of pre-vaccine and post-H1N1 vaccination sera from two individuals with different neutralizing antibody titers (in parenthesis) is shown with recombinant mammalian H1N1 HA0 in (E) and properly folded bacterially expressed H1N1 HA1 (1–330) in (F) or H1N1 HA (1–480) in (G). Binding was recorded using ProteOn system surface plasmon resonance biosensor instrument (BioRad Labs, Hercules, CA).

### Properly folded bacterial H1N1 HA proteins adsorb neutralizing activity in post-H1N1 vaccination and post-H1N1 infection sera

The functional relevance of binding to properly folded bacterially expressed H1N1-HA proteins was further confirmed in adsorption experiments (Table 1). Both bacterially expressed HA1 (1–330) and HA (1–480) proteins and the mammalian cell derived HA0 adsorbed most of the neutralizing activity of H1N1 hyperimmune sheep sera (NIBSC), reducing the MN titer from 1∶6,400 to <1∶40 (Table 1, top panel). Similar results were obtained with post-H1N1 infection ferret sera from day 21. The H1N1-HA1 (1–330) reduced the neutralizing activity of the convalescent sera from 1∶1,280 to <1∶40. In the case of HA0 (mammalian) and bacterial HA (1–480), residual neutralizing activity (1∶80) was observed after sera adsorption (Table 1, lower panel).

**Table 1:** Adsorption of neutralization activity using HA proteins.

Sheep anti-A/California/07/2009 -HA-sera (NIBSC)	
Peptides added	TITER*
No peptide	6400
HA 1–330 - FLOW-THROUGH	<40
HA 1–480 - FLOW-THROUGH	<40
Mammalian HA0 - FLOW-THROUGH	<40
GST-His - FLOW-THROUGH	6400

Ferret anti-A/California/07/2009 -infected sera	
No peptide	1280
HA 1–330 - FLOW-THROUGH	<40
HA 1–480 - FLOW-THROUGH	80
Mammalian HA0- FLOW-THROUGH	80
GST-His - FLOW-THROUGH	1280

*End-point titers (mean of three replicates) using polyclonal rabbit sera in a microneutralization assay performed with A/California/07/2009 (X-179A).

The combined data from the CD melt, SPR-based binding assays, and adsorption studies demonstrated that both bacterially expressed proteins are properly folded and express antigenically relevant conformational neutralizing epitopes. However, only the HA1 globular domain but not the HA ectodomain (or the mammalian cell expressed HA0) contained functional trimers and oligomers required for fetuin binding and RBC agglutination.

### Immunization of rabbits and sheep with bacterially expressed H1N1 HA1 (1–330) and HA (1–480) and mammalian HA0 proteins

To evaluate the immunogenicity of the bacterially expressed proteins, we immunized rabbits after mixing of HA1 (1–330) or HA (1–480) with Titermax adjuvant. The pre- and post vaccination sera were evaluated by microneutralization assay. Even after a single immunization with HA1 (1–330), rabbits had a MN titer of 1∶40. After second and third immunizations high MN titers were measured (6,400 and 25,600, respectively) (Table 2, top panel). The HA (1–480) elicited H1N1 neutralizing antibodies only after the second and third boosts, and the peak MN titers (3,200 and 6,400, respectively) were lower compared with the HA1 (1–330) immunized rabbits. In a separate study, sheep were vaccinated with mammalian derived HA0 (Immune Technology Corps) or with the bacterially–expressed HA1 (1–330) (Table 2, bottom panels). Again, the kinetics of immune responses and the peak neutralization titers were significantly higher for the sheep immunized with the bacterially-expressed HA1 (1–330) protein compared with the mammalian HA0 expressed and purified from 293 cells.

**Table 2:** Mean reciprocal neutralizing titers of Rabbit and Sheep anti-HA sera.

RABBIT	SERA	END-POINT TITERS*
**H1N1-HA (1–330)**	Pre Vaccine	<20
	Post- 1	**40**
	Post- 2	**6,400**
	Post- 3	**25,600**
**H1N1-HA (1–480)**	Pre Vaccine	<20
	Post- 1	<20
	Post- 2	**3,200**
	Post- 3	**6,400**
**SHEEP**		
**Mammalian H1N1-HA0**	Pre Vaccine	<20
	Post- 1	<20
	Post- 2	**1,600**
	Post- 3	**6,400**
**H1N1-HA (1–330)**	Pre Vaccine	<20
	Post- 1	**80**
	Post- 2	**12,800**
	Post- 3	**51,200**

*End-point titers (mean of three replicates) using polyclonal rabbit sera in a microneutralization assay performed with A/California/07/2009 (X-179A).

### Vaccination and challenge studies in ferrets

The protective immunity elicited by bacterially expressed proteins was further evaluated in a ferret challenge model [25]. Female Fitch ferrets (*n* = 4 in each group) were vaccinated intramuscularly in the quadricep muscle on day 0 and boosted on day 21 with either HA1 (1–330) or HA (1–480) proteins at 7.5 and 30 μg dose combined with Titermax adjuvant. Serum samples were collected after vaccinations and analyzed in HAI (Fig. 3). The 30 μg dose induced 2–4 fold higher titers compared with the 7.5 μg dose for both bacterially expressed proteins (Fig. 3). However, at the lower dose of 7.5 μg, the HA1 (1–330) consistently elicited higher HAI titers compared with the HA (1–480) at the same dose. The observed HAI titers measured in the current study were similar to data from recently reported ferret vaccination studies in which commercially available live attenuated or split-inactivated licensed vaccines were used [26], [27].

**Figure 3:** Hemagglutination-inhibition (HAI) titers in ferrets. HAI antibody in ferrets (*n* = 4 per group) vaccinated with either 30 µg or 7.5 µg of influenza H1N1 HA1 or HA. Blood was collected at day 35 (post-dose 2). HAI responses were assessed against A/California/07/2009. Bars indicate geometric mean titer (GMT). The titer from each individual ferret is indicated by symbol. *p = 0.05 HA (1–480) low dose vs. HA (1–480) high dose.

Following second vaccination, ferrets were challenged intranasally with 1×10^6^ 50% egg infectious doses (EID_50_) (∼1×10^5.75^ TCID_50_/ml) of A/California/07/2009 virus in a volume of one milliliter. To determine viral loads in nasal washes, each ferret was administered each day post-challenge with 1.5 ml of 0.9% saline to each nare and washes were collected for virus titer determinations using the plaque assay.

In unvaccinated animals (naïve), viral loads in the nasal washes were highest on day 1, gradually declining on days 3 and 5 (Fig. 4A) and were back to baseline on day 7 as previously described[25]. Among the vaccinated animals, the high dose groups (30 μg), receiving either HA1 (1–330) or HA (1–480), reduced viral titers by >2 logs as early as day 1 post challenge. In the 7.5 μg vaccinated animals, virus replication on day 1 was observed, followed by a more rapid decline compared with the unvaccinated animals (Fig. 4A). Between day 3 and 5, a more rapid virus clearance was observed in the HA1 (1–330) vaccinated groups compared with the HA (1–480) vaccinated group or the naïve group (Fig. 4A).

**Figure 4:** Viral loads and morbidity following A/California/07/2009 challenge in ferrets. (**A**) **Viral replication of influenza A/California/07/2009 in nasal washes following intranasal challenge.** Average pfu of virus from the nasal washes of each group (4 ferrets per group) on days 1, 3, and 5 post challenges. (B) **Change in body temperature and** (**C**) **percent body weight.**

In terms of morbidity, sustained elevation in body temperatures were measured in the naïve group post H1N1 virus challenge between days 1–4 (Fig. 4B). Inactivity and weight loss were also recorded up to day 7, followed by a slow recovery that did not reach normal weights by day 13 (termination) (Fig. 4C and data not shown). The HA1 (1–330) vaccinated animals that received 30 μg protein showed no temperature elevation and no weight loss (Fig. 4B-C). The 7.5 μg HA (1–330) vaccine dose also showed no weight loss and only a brief mild increase in body temperature on Day 2 (Fig. 4B-C). The HA (1–480) vaccinated animals at the 30 μg dose also showed no weight loss, and a transient elevation in body temperature on days 1–3 (not as high as in the naive group). But the animals that received HA (1–480) at the lower dose (7.5 μg) showed an increase in body temperature similar to the naïve group and some weight loss on days 2–6 post challenge.

Together, these data demonstrate that properly folded bacterially expressed unglycosylated H1N1 HA proteins, elicited high neutralizing antibody titers in ferrets, not different from previously reported antibody responses against licensed influenza vaccines ([26], [27]. Importantly, at the lower vaccine dose of 7.5 μg, the HA1 (1–330) that contained both trimers and oligomers protected ferrets from morbidity more efficiently than the HA (1–480), which only contain monomers. The clinical symptoms correlated with the observed HAI titers prior to challenge.

## Discussion

The recent 2009-H1N1 swine-like virus influenza pandemic highlighted the need to rapidly produce enough vaccine doses for global vaccination brought to light the shortcomings of the traditional process of manufacturing influenza vaccines and the need to use alternative approaches for a more rapid generation of vaccine for global immunization in response to impending influenza pandemic. Bacterially expressed HA proteins can be manufactured rapidly and are amenable to mass production that can fulfill global vaccine needs. The main challenge to the prokaryotic production system is to ascertain proper refolding of expressed HA proteins representative of native HA spike structures on influenza virus. In addition to properly folded HA monomers, higher MW structures (*i.e.,* trimers and oligomers) are important and likely to contribute to the optimal immunogenicity of the HA, since all influenza neutralizing antibodies are conformation dependent and some trimer specific antibodies have potent neutralizing activity [28]. In eggs and mammalian cells, post-translational glycosylation contribute to the proper folding, trimerization and transport of the newly synthesized HA molecules to the cell membrane [18]. However, in the case of recombinant HA proteins, trimerization is not always found even in eukaryotic cell substrates [11].

The main findings in the current study are: (a) bacterially expressed H1N1 HA1 (1–330) and HA (1–480) can be purified as properly folded proteins as determined by CD spectroscopy, SPR analyses with H1N1 immune sera, and adsorption of neutralizing activity from post-infection and post vaccination sera; (b) the HA1 (1–330) contained >50% trimeric and oligomeric forms and could bind to fetuin and agglutinated human RBC, while the HA (1–480) and mammalian cell expressed HA0 proteins were predominantly monomeric, did not bind fetuin, and did not agglutinate RBC; (c) the HA1 (1–330) induced higher titers of neutralizing antibodies compared with HA (1–480) or mammalian derived recombinant HA0 in rabbits and sheep; (d) in a ferret H1N1 challenge model, high-dose vaccination (30 μg HA) with both bacterially expressed HA1 (1–330) and HA (1–480) proteins protected animals from morbidity (elevated body temperature and weight loss) following challenge with novel H1N1 A/California/07/2009 virus. However, low-dose vaccination (7.5 μg HA) of ferrets with HA1 (1–330) resulted in lower morbidity and more rapid virus clearance compared with the HA (1–480) vaccinated group.

This study extends our previous reports with the H5N1 highly pathogenic virus, in which we have used whole-genome-phage display libraries (GFPDL) to map the antibody responses following human infection or vaccination. We have identified large HA1 fragments, encompassing the receptor binding domain (RBD), that were bound by broadly neutralizing human monoclonal antibodies from H5N1 recovered individuals and by their polyclonal convalescent sera [12]. In a subsequent study, we found that following vaccination with inactivated H5N1 (A/Vietnam/1203/2004) influenza vaccine the immune sera from the MF59-adjuvanted vaccinated individuals bound with much higher avidity to bacterially expressed properly folded H5 HA1 proteins compared with unadjuvanted vaccine sera [13]. Importantly, the bacterially expressed HA1 proteins were also shown to absorb most of the neutralizing activity in post infection and post vaccination sera [12], [13]. Based on these studies, we hypothesized that bacterially-expressed HA1 fragments if properly folded, could be useful as vaccines against emerging influenza strains.

In the current study, we found that expression and purification of properly folded H1N1 HA1 (1–330) (lacking HA2) in bacterial system was more efficient and gave higher yield compared with the larger HA ectodomain (1–480). Between 39–45 mg of >90% purified HA1 (1–330) protein can be obtained from 1 liter of bacterial batch culture, while the yield for HA (1–480) was only 0.4–0.8 mg/L. In addition to the much lower yield, the HA (1–480) contained only monomers, and as a result, it did not bind to fetuin and did not agglutinate RBC. Both of these functions require the presence of quartenary HA forms (i.e. trimers and oligomers). Mammalian expressed HA0 protein exhibited the same properties as the bacterially expressed HA(1–480) ectodomain. This is in agreement with previous reports on full length HA ectodomain proteins expressed in a variety of cell substrates wherein peptide linkers were introduced to facilitate oligomerization [11]. Similar to our findings, the oligomerized cell-based HA product showed better neutralizing antibodies than its monomeric counterpart [11].

While both proteins were immunogenic in ferrets at the high dose of 30 μg, the HA1 (1–330) was more immunogenic and protected ferrets from H1N1 morbidity more efficiently at a lower dose (7.5 μg) compared with the HA (1–480) protein. In the case of mass vaccination, dose sparing is likely to be of great impact.

The ability of HA1 globular domain to form trimers has not been reported before. We have recently confirmed that bacterially expressed HA1 globular heads from multiple influenza strains (avian H5N1 and seasonal strains), can be produced at high yield. In all cases the HA1 proteins contain trimers and oligomers and agglutinate RBC. Studies to map the trimerization signal of HA1 are ongoing.

In the face of an impending influenza pandemic, HA1 proteins derived from the newly spreading virus can be rapidly expressed in bacterial systems several months before the traditional approach using vaccine strains generated via either gene reassortment or reverse genetics, followed by adaptation to growth in eggs. With appropriate testing methods in place to monitor proper folding and biological activity (hemagglutination assay), this simple and efficient approach may provide an early vaccine for large scale production to fulfill global vaccine needs in a much shorter time frame. Moreover, bacterially produced HA vaccines may also be an alternative for humans with known egg allergies that cannot be immunized with traditional influenza vaccines produced in eggs.

## Materials and Methods

### Expression vector and cloning of H1N1-HA1 (1–330) and HA (1–480)

cDNA corresponding to the HA gene segment of A/California/07/2009 was generated from RNA isolated from egg-grown virus strain, and was used for cloning. pSK is a T7 promoter based expression vector where the desired polypeptide can be expressed as fusion protein with His_6_ tag at the C-terminus. DNA encoding HA1 (1–330) and HA (1–480) were cloned as *Not*I-*Pac*I inserts in the pSK expression vector.

### Protein expression, refolding and purification

*E. coli* Rosetta Gami cells (Novagen) were used for expression of H1N1-HA1 (1–330) and HA (1–480). Following expression, inclusion bodies (IB) were isolated by cell lysis and multiple washing steps with 1% Triton X-100. The final IB pellets were resuspended in denaturation buffer containing 6M Guanidine Hydrochloride and dithioerythreitol (DTE) at final protein concentration of 10 mg/ml, and were centrifuged to remove residual debris. For refolding, supernatants were slowly diluted 100-fold in redox folding buffer [13]. The renaturation protein solution was dialyzed against 20 mM Tris HCl pH 8.0 to remove the denaturing agents. The dialysates were filtered through 0.45 μm filters, and were subjected to purification by HisTrap Fast flow chromatography. This process was previously shown to generate highly purified properly folded HA1 fragments from H5N1 [13].

### Circular Dichroism (CD)-monitored equilibrium unfolding experiment

To demonstrate that the bacterially expressed HA fragments are properly folded they were analyzed by CD spectroscopy [13]. For CD spectroscopy in solution, H1N1-HA proteins were dissolved in 20 mM PBS, pH 7.4, at 0.1 mg/ml. The change in elipticity at 222 nm (to follow unfolding of α-helices) during unfolding was monitored using a J-715 Circular Dichroism system (JASCO). The unfolding reaction was initiated by subjecting the protein in PBS to 1°C/min increments. The experiments were carried out in triplicate.

### Gel filtration Chromatography

H1N1-HA1 (1–330) and HA (1–480) at a concentration of 5 mg/ml were analyzed on Superdex S200 XK 16/60 column (GE-Healthcare) pre-equilibrated with PBS, and the protein elution monitored at 280 nm. Protein molecular weight marker standards (GE healthcare) were used for column calibration and generation of a standard curve to identify the molecular weights of the test protein sample.

### Affinity measurements by surface plasmon resonance

Steady-state equilibrium binding of post-H1N1 vaccine or post-H1N1 infection sera was monitored at 25°C using a ProteOn surface plasmon resonance biosensor (BioRad Labs). The H1N1-HA proteins were coupled to a GLC sensor chip (BioRad Labs) with amine coupling with 500 resonance units (RU) in the test flow cells. Ten-fold dilution of animal sera (60 µl) was injected at a flow rate of 30 µl/min (120-sec contact time). Flow was directed over a mock surface to which no protein was bound, followed by the HA protein coupled surface. Responses from the protein surface were corrected for the response from the mock surface and for responses from a separate, buffer only, injection. MAb 2D7 (anti-CCR5) and naïve ferret sera were used as a negative control antibody in the experiments. Binding kinetics for the animal sera and the data analysis were performed with BioRad ProteON manager software (version 2.0.1). Similar binding studies were previously conducted with H5N1 HA1 proteins. Human monoclonal antibodies with conformation-dependent epitopes bound only to the properly folded HA proteins that were purified at pH 7.2 (identical to the current study) but not to unfolded HA1 proteins, purified at pH 3.0 [13].

### Receptor binding assay using surface plasmon resonance

Binding of different HA1 derivatives to fetuin (natural homolog of sialic acid cell surface receptor proteins) and its asialylated counterpart (Asialo-fetuin) was analyzed at 25°C using a ProteOn surface plasmon resonance biosensor (BioRad Labs). Fetuin or Asialo-fetuin (Sigma) were coupled to a GLC sensor chip with amine coupling at 1000 resonance units (RU) in the test flow cells. Samples of 60 µl freshly prepared H1N1-HA1, HA0, and mammalian derived HA0 proteins at 10 µg/ml were injected at a flow rate of 30 µl/min (120-sec contact time). Flow was directed over a mock surface to which no protein was bound, followed by the fetuin or asialo-fetuin coupled surface. Responses from the protein surface were corrected for the response from the mock surface and for responses from a separate, buffer only, injection. Binding kinetics and data analysis were performed with BioRad ProteON manager software (version 2.0.1).

### Hemagglutination Assay

Human erythrocytes were separated from whole blood (Lampire Biologicals). After isolation and washing, 30 µl of 1% human RBC suspension (vol/vol in 1% BSA-PBS) was added to 30 µl serial dilutions of HA protein or influenza virus in 1% BSA-PBS in a U-bottom 96-well plate (total volume, 60 µl). Agglutination was read after incubation for 30 min at room temperature.

### Neutralizing Antibodies Adsorption with HA proteins

Five-fold diluted post-H1N1 vaccination (NIBSC) sera or post-H1N1 infection ferret sera (500 µl) were added to 0.5 mg of purified HA-His_6_ or to control GST-His_6_ protein, and incubated for 1 hr at RT. Nickel-nitrilotriacetic acid (Ni-NTA) magnetic beads (200 µl) (Qiagen) were added for 20 min at RT on end-to-end shaker, to capture the His-tagged proteins and the antibodies bound to them, followed by magnetic separation. Supernatants containing the unbound antibodies were collected. The pre-and post-adsorbed sera were subjected to virus microneutralization assay.

### Rabbit immunization and virus neutralization assays

White New Zealand rabbits were immunized three times intramuscularly at 21-day intervals with 100 µg of purified H1N1-HA1 (1–330) or HA 1–480) proteins with Titermax adjuvant (Titermax Inc). Virus-neutralizing titers of pre- and post vaccination rabbit sera were determined in a microneutralization assay based on the methods of the pandemic influenza reference laboratories of the Centers for Disease Control and Prevention (CDC). Low pathogenicity H1N1 virus, generated by reverse genetics, was obtained from CDC (X-179A). The experiments were conducted with three replicates for each serum sample and performed at least twice.

### Vaccination of ferrets and blood collection

Ferrets used in the study were tested to be sero-negative for circulating seasonal influenza A (H1N1 and H3N2) and influenza B viruses by HAI. Female Fitch ferrets (*n* = 4 in each group) were vaccinated intramuscularly in the quadriceps muscle on day 0 and boosted on day 21 and then challenged with virus on day 35. Control animals (*n* = 4) were mock vaccinated with phosphate buffered saline (PBS; pH 7.2). Each animal was vaccinated with one of two doses (30 μg or 7.5 μg) of recombinant HA in sterile 0.9% saline. Each vaccine was mixed with the adjuvant formulation, TiterMax (TiterMax USA, Inc, Norcross, Georgia, US) at a 1∶1 ratio. The volume for all intra-muscular vaccinations was 0.5 ml. The first and second vaccinations were given in the left and right hind legs, respectively. Blood was collected from anesthetized ferrets via the anterior vena cava. The collected blood was transferred to a tube containing a serum separator and clot activator and allowed to clot at room temperature. Tubes were centrifuged at 6000 rpm for 10 minutes; serum was separated, aliquoted and stored at −80±5°C. All procedures were in accordance with the National Research Council (NRC) Guidelines for the Care and Use of Laboratory Animals, the Animal Welfare Act, and the Centers for Disease Control (CDC)/National Institutes of Health (NIH) Bio- Safety Guidelines in Microbiological and Biomedical Laboratories and approved by the Institutional Animal Care and Use Committee (IACUC).

### Infection and monitoring of Ferret

Animal experiments with virus A/California/07/2009 were performed in the AALAC-accredited ABSL-3 enhanced facility. Animals were infected and monitored as previously described[27] except using 5% isofluorane anesthesia. Briefly, ferrets were anesthetized with isofluorane and infected intranasally with 1×10^6^ 50% egg infectious doses (EID_50_) (∼1×10^5.75^ TCID_50_/ml) of A/California/07/2009 in a volume of one milliliter. Animals were monitored for temperature, weight loss, loss of activity, nasal discharge, sneezing and diarrhea daily following viral challenge. To determine viral load from nasal washes, 1.5 ml of 0.9% saline was administered to each nare and the wash was collected each day post-challenge of each ferret. Temperatures were measured through use of an implantable temperature transponder (BMDS, Sayre, PA) and were recorded at approximately the same time each day. Pre-infection values were averaged to obtain a baseline temperature for each ferret. Clinical signs of sneezing and nasal discharge, inappetence, dyspnea, neurological signs, respiratory distress, and level of activity were assessed daily. A scoring system was used to assess activity level where 0  =  alert and playful; 1  =  alert but playful only when stimulated; 2  =  alert but not playful when stimulated; 3  =  neither alert nor playful when stimulated. Based on the daily scores for each animal in a group, a relative inactivity index was calculated [29].

### Hemagglutinination Inhibition (HAI) assay

RDE-treated ferret sera were serially diluted in v-bottom 96-well microtiter plates followed by the addition of 8 hemagglutination units (HAU) of influenza virus. Following an incubation of approximately 20 minutes, 0.5% suspension of turkey RBC (TRBC) in PBS (pH 7.2) were added and mixed by agitation. The TRBCs were allowed to settle for 30 minutes at room temperature and HAI titers were determined by the reciprocal value of the last dilution of sera which completely inhibited hemagglutination of TRBC. A negative titer was defined as 1∶10.

### Determination of viral loads

Viral loads in nasal washes were determined by the plaque assay. Briefly, MDCK cells plated in 6-well tissue culture plates were inoculated with 0.1 ml of virus-containing sample, serially diluted in Dulbecco's modified Eagle's medium (DMEM). Virus was adsorbed to cells for 1 h, with shaking every 15 min. Wells were overlaid with 1.6% w/v Bacto agar (DIFCO, BD Diagnostic Systems, Palo Alto, CA, USA) mixed 1∶1 with L-15 media (Cambrex, East Rutherford, NJ, USA) containing antibiotics and 0.6 mg/ml trypsin (Sigma, St. Louis, MO, USA). Plates incubated for 5 days. Cells were fixed for 10 minutes using 70% v/v Ethanol and then overlaid with 1% w/v crystal violet. Cells were then washed with deionized water to visualize plaques. Plaques were counted and compared to uninfected cells.
